RETRACTED

# ANLN Regulated by miR-30a-5p Mediates Malignant Progression of Lung Adenocarcinoma

**DOI:** 10.1155/2021/9549287

**Published:** 2021-11-05

**Authors:** Feng Deng, Zhili Xu, Jun Zhou, Ruhu Zhang, Xiaowei Gong

**Affiliations:** Department of Thoracic Surgery, Jiangyin Hospital of Traditional Chinese Medicine, Jiangyin Hospital Affiliated to Nanjing University of Chinese Medicine, Jiangyin 214400, China

## Abstract

**Background:**

ANLN and miR-30a-5p may be involved in the progression of lung adenocarcinoma (LUAD). However, their underlying mechanism in LUAD has not been completely comprehended.

**Methods:**

Differential expression analysis, binding site prediction, and survival analysis were conducted by bioinformatics approaches. ANLN mRNA and miR-30a-5p expression were detected by qRT-PCR. ANLN protein expression was detected by western blot. Cell behaviors in LUAD were examined by functional experiments.

**Results:**

ANLN was activated in LUAD cells in terms of mRNA and protein. High ANLN level was positively correlated with poor prognosis. Enforced ANLN stimulated protumorigenesis LUAD cell behaviors. miR-30a-5p could target ANLN mRNA, as revealed and verified through assays. Remarkably low miR-30a-5p expression was observed in LUAD cells, and it could repress ANLN expression. The accelerated cell behaviors by overexpression of ANLN were counteracted by upregulating miR-30a-5p.

**Conclusion:**

Overall, miR-30a-5p remarkably restrained the malignant progression of LUAD cells by constraining ANLN expression. Thus, ANLN and miR-30a-5p could be novel therapeutic targets of LUAD.

## 1. Introduction

Lung cancer is an unbearably painful illness as well as a fetal tumor [1]. Missed diagnosis in its early-stage triggers poor prognosis of patients [2]. Lung adenocarcinoma (LUAD) is a prevalent subtype of lung cancer which kills millions of people all over the world [3]. Characterized by tumor metastasis to nearby or distant organs, treatment for such advanced disease faces a great challenge. Nevertheless, molecular mechanism related to the metastasis of LUAD has not been fully clarified, and a better understanding of the mechanism can help to improve therapy on patients.

Anillin (ANLN), located on chromosome 7p14.2 first found in fruit flies, encodes actin-binding proteins [4]. In normal tissues, ANLN level is activated in placenta, cerebrum, and testis while it is relatively low in other tissues [5]. As several references uncovered, ANLN is aberrantly expressed in many cancers like cervical cancer [6], breast cancer [7], pancreatic cancer [8], prostatic cancer [9], and anaplastic thyroid carcinoma [10]. Besides, inactivating ANLN restrains cell growth in NSCLC while the overexpression of ANLN can promote the cell movement [11]. So far, a study has reported that ANLN participates in cell developmental processes via regulating nuclear division pathway in LUAD [12]. Moreover, activation of ANLN hastens epithelial-mesenchymal transition (EMT) of tumor cells [13]. Nevertheless, far less has been illustrated on regulatory role of ANLN in LUAD.

RETRACTED

MicroRNAs (miRNAs) are capable of mediating levels of relevant mRNAs [14, 15]. miR-30a-5p is involved in the development of a wide range of tumors, such as esophageal squamous cell carcinoma [16], pancreatic ductal adenocarcinoma [17], prostatic cancer [18], and colorectal cancer [19]. Abnormally-expressed miR-30a-5p in NSCLC can repress EMT process of cancer cells [20, 21]. Moreover, miR-30a-5p is mediated by LINC00461 in NSCLC, in turn, affecting the level of ZEB2 to influence tumor progression [22]. However, much more molecular mechanisms of miR-30a-5p should be studied in LUAD.

Thus, we found by bioinformatics analysis that levels of ANLN and miR-30a-5p were in connection with prognosis of LUAD patients. Besides, we also evaluated the influence of overexpressed ANLN or miR-30a-5p on LUAD cell functions.

## 2. Materials and Methods

### 2.1. Bioinformatics Approaches

Expression data of mature miRNA (Normal: 46, Tumor: 521) and mRNA (normal: 59, tumor: 535) were firstly accessed from the TCGA-LUAD dataset (https://portal.gdc.cancer.gov/). The “edgeR” package was used to analyze the differential expression of miRNAs and mRNAs (∣logFC | >1.5, *p*adj < 0.05). The mRNA of interest was chosen for research after searching references. miRNAs potentially targeting the interested mRNA were predicted via TargetScan (http://www.targetscan.org/vert_72/), miRDB (http://mirdb.org/), and starBase (http://starbase.sysu.edu.cn/) databases, and then the predicted miRNAs were intersected with the differentially expressed miRNAs. At last, the highest correlated miRNA with the mRNA was selected via Pearson correlation analysis for further research.

### 2.2. Cell Culture and Transfection

Human normal lung epithelial cell line BEAS-2B (BNCC100240) and human LUAD cell line PC9 (BNCC340767) were maintained in Dulbecco's modified Eagle medium (DMEM) (BNCC351841, BNCC, China) with 10% fetal bovine serum (FBS). Human LUAD cell line A549 (BNCC337696) was maintained in F-12K medium (BNCC341829, BNCC, China) containing 10% FBS. Human LUAD cell lines H1299 (BNCC100268) and H1975 (BNCC340345) were incubated in RPMI-1640 medium (BNCC341471, BNCC, China) plus 10% FBS. Culture conditions were 5% CO_2_ and 37°C. miR-30a-5p mimic and mimic NC (mirVana™ miRNA Mimic, negative control #1, 4464058) were synthesized by Thermo Fisher Scientific (USA). pcDNA3.1-ANLN plasmid (oe-ANLN), pcDNA3.1 control plasmid (oe-NC), ANLN siRNA (si-ANLN), and ANLN siRNA control (si-NC) were synthesized by GenePharma (Shanghai, China). For cell transfection, Lipofectamine™ 2000 (Invitrogen, USA) was introduced. Briefly, cells were cultivated in 6-well plates (Thermo Fisher, Waltham, USA) until transfection. 4 *μ*g plasmids or 100 nM miRNA mimic was added into each construct followed by 24 h incubation.

RETRACTED

### 2.3. Quantitative Real-Time PCR (qRT-PCR)

The TRIzol (Invitrogen, Carlsbad, CA, USA) was employed to extract total RNA. ReverTra Ace qRT-PCR kit (Toyobo, Osaka, Japan) was used for RNA reverse transcription to acquire cDNA. qRT-PCR was performed on the products with THUNDERBIRD SYBR® qPCR Mix (Toyobo, Osaka, Japan). PCR procedures were predenaturation at 94°C for 2 min, denaturation at 94°C for 30 sec, annealing at 56°C for 30 sec, extension at 72°C for 1 min, repeat the previous procedure for 30 times, and continuous extension at 72°C for 10 min. U6 and *β*-actin were selected as internal references for miR-30a-5p and ANLN, respectively. Results were shown by 2^-*ΔΔ*Ct^ value. Primer sequences are presented in Table 1.

### 2.4. CCK-8 Analysis

Cell proliferation was detected with colorimetric determination method. Cell counting kit-8 (CCK-8; Dojindo Molecular Technologies, Inc., Japan) was employed to measure cell viability. In detail, cells were seeded into 96-well plates (10^4^ cells per well) after 24 h of transfection. After culturing for 0, 24, 48, 72, and 96 h, 10 *μ*L CCK-8 reagent was added into each well for another 1 h of incubation at 37°C, respectively. At last, absorbance was recorded at 490 nm.

### 2.5. Wound Healing Assay

LUAD cell line A549 was incubated in 6-well plates at 2 × 10^5^ cells per well. When cell coverage reached to about 80%, 100 *μ*L sterilized micropipette tip was used to scrape well surface, after which PBS was used for washing, followed by cell incubation in the medium containing 2% FBS. Finally, cell migration status at 0 and 24 h was observed by a microscope and photographed.

### 2.6. Transwell Assay

The upper Transwell chambers were coated by Matrigel (356234, BD Company, USA, 20 *μ*L,0.5 g/L), and the Matrigel was balanced for 20 min in an incubator. Cells that were transfected for 24 h were collected to make 200 *μ*L cell suspension which was then added into the upper chambers, and medium with 10% FBS was added into the lower chambers. After incubation for 36 h, the cells failing to pass through the Matrigel membrane were removed, and the invaded cells were fixed in 4% paraformaldehyde followed by staining with 0.1% crystal violet. The number of stained cells was counted by microscopy in several randomly selected fields, and the average numbers in each field were recorded.

RETRACTED

### 2.7. Western Blot (WB)

Total proteins were obtained from cell lysates by RIPA lysis buffer (Beyotime, Shanghai, China) and quantified with the Pierce BCA protein assay kit (Pierce, Rockford, IL, USA). Next, 10 *μ*g proteins were subjected to sodium dodecyl sulfate polyacrylamide gel electrophoresis under 200 mA constant current and then transferred on a PVDF membrane within 120 min. Later, the membrane was blocked using 5% skim milk for 2 h, followed by incubating with primary antibodies mouse anti-ANLN (1 : 500, ab211872, Abcam, UK) and mouse anti-*β*-actin (1 : 10000, ab6276, Abcam, UK) at 4°C overnight. Next, the membrane was rinsed with TBST for 3 times and added with secondary antibody goat anti-mouse IgG H&L (HRP) (1 : 10000, ab205719, Abcam, UK) for 1 h of incubation. Protein bands were presented with the enhanced chemiluminescence (ECL Plus) detection system (Thermo Scientific) and analyzed with Image Lab.

### 2.8. Dual-Luciferase Assay

Sanger sequencing was applied to determine wild-type (WT) and mutant (MUT) ANLN 3′UTR sequences, and then the sequences were inserted into pmiRGLO luciferase miRNA target expression vectors (Promega). Next, the obtained vectors (ANLN-WT and ANLN-MUT) were cotransfected with miR-30a-5p mimic/mimic NC into LUAD cell line A549 which had been cultured at 37°C for 24 h. After culture for 48 h, the luciferase detection reagent (Promega, Fitchburg, WI, USA) was used to determine luciferase activity.

### 2.9. Data Analysis

GraphPad Prism 6.0 was applied to statistically analyze the results and make figures. Results were represented in a manner of mean ± SD. Two-group differences were analyzed by *t* test, and multigroup differences were analyzed by one way analysis of variance. *p* < 0.05 denoted statistically significant. Each assay experienced 3 repetitions.

## 3. Results

### 3.1. Markedly Activated ANLN in LUAD Cells Indicates Poor Prognosis

The results of edgeR differential analysis showed 3,611 differential mRNAs (Figure 1(a)). References have illustrated that ANLN is activated in various cancer tissues and involved in carcinogenesis [23, 24]. Therefore, we selected ANLN for research. First, expression data of mRNAs downloaded from the TCGA-LUAD dataset indicated that the ANLN level in normal tissues was remarkably lower than that in LUAD tissues (Figure 1(b)). Besides, patients with highly expressed ANLN had poor prognosis (Figure 1(c)). Moreover, the correlations between clinicopathological features and ANLN expression were analyzed, whose results revealed a relatively high level of ANLN in patients with lymph node metastasis and advanced stage (Figure 1(d)). qRT-PCR and WB revealed that compared with normal cells, LUAD cells displayed conspicuous increased mRNA and protein of ANLN, and level of ANLN was the highest in A549 cell line (Figures 1(e) and 1(f)). These results revealed that activated ANLN was positively correlated with poor prognosis, lymph node metastasis, and advanced stage. Thus, we chose the A549 cell line for the following experiments.

RETRACTED

### 3.2. Overexpressing ANLN Promotes Progression of LUAD Cells

To determine whether ANLN could influence cell progression in LUAD, the expression of ANLN was modulated by transfecting oe-ANLN and si-ANLN vectors into the A549 cell line. qRT-PCR uncovered that ANLN level in the oe-ANLN and si-ANLN groups was markedly elevated and decreased, respectively (Figure 2(a)), which indicated that ANLN was successfully overexpressed and downregulated. CCK-8 assay represented that cells in the oe-ANLN group had greatly increased proliferative ability, while this ability was suppressed upon si-ANLN treatment (Figure 2(b)). Moreover, Transwell assay testified that overexpressed ANLN increased the invasive ability of cells, while this ability was restrained upon si-ANLN treatment (Figure 2(c)). It is established that smaller wound healing area manifests weaker migratory ability. Wound healing area was significantly increased in the oe-ANLN group, thus, the migratory ability of cells in the ANLN overexpressed group was stronger, where this ability was weakened upon si-ANLN treatment (Figure 2(d)). Hence, we held the belief that upregulated ANLN could promote the progression of LUAD.

### 3.3. Conspicuously Low Level of miR-30a-5p in LUAD Cells

Considering that the expression of mRNA in cancers would be regulated by miRNAs, we kept on digging the upstream miRNA which would be involved in the regulation of ANLN on the progression of LUAD to improve related functional mechanism. Totally, 186 differential miRNAs were obtained through differential analysis based on miRNA data collected from the TCGA database (Figure 3(a)). Then, the 39 downregulated differential miRNAs were intersected with the upstream regulator miRNAs of ANLN predicated by public databases, by which 3 differential miRNAs (miR-30a-5p, miR-195-5p, and miR-374b-5p) potentially targeting ANLN were acquired (Figure 3(b)). Pearson correlation analysis revealed the highest negative correlation coefficient between miR-30a-5p and ANLN (Figure 3(c)). Besides, TCGA-LUAD data showed a lower miR-30a-5p expression in tumor tissues than that in normal tissues (Figure 3(d)). Hence, miR-30a-5p was selected for the in-depth study below. Further analysis of miR-30a-5p expression in different cell lines was conducted, by which a lower expression of miR-30a-5p in four LUAD cell lines was observed (Figure 3(e)).

RETRACTED

### 3.4. miR-30a-5p Constrains ANLN in LUAD

We firstly predicted the binding site between ANLN and miR-30a-5p via bioinformatics databases (Figure 4(a)). In the meantime, ANLN-WT/MUT vectors and miR-30a-5p mimic/mimic NC were cotransfected into A549 cells for dual-luciferase reporter gene detection. It was uncovered that the luciferase activity in the ANLN-WT group was evidently suppressed with overexpression of miR-30a-5p, suggesting that miR-30a-5p was directly bound to ANLN (Figure 4(b)). Through qRT-PCR and WB, we testified that ANLN expression was considerably hampered in miR-30a-5p overexpressed group in the A549 cell line compared to the control group (Figures 4(c) and 4(d)). Thus, we speculated that ANLN was the target gene of miR-30a-5p.

### 3.5. Upregulating miR-30a-5p Can Reverse the Promoting Effect of ANLN Upregulation on LUAD Cell Activities

Three kinds of cell lines, normal A549 cell line (miR-NC), pcDNA3.1-ANLN transfected A549 cell line (miR-NC + oe-ANLN), and miR-30a-5p mimic/pcDNA3.1-ANLN transfected A549 cell line (miR-mimic+oe-ANLN), were constructed. The increased expression levels of ANLN mRNA and protein in the miR-NC + oe-ANLN group were found to be greatly recovered in the miR-30a-5p mimic+oe-ANLN group via qRT-PCR and WB (Figures 5(a) and 5(b)). CCK-8 assay was performed to detect the proliferative ability of LUAD cells, whose results illustrated that the proliferative ability of LUAD cells was remarkably strengthened in the miR-NC + oe-ANLN group, while the ability was weakened after miR-30a-5p was simultaneously overexpressed (Figure 5(c)). Afterward, Transwell assay and wound healing assays indicated the enhanced abilities of A549 cell invasion and migration by overexpressing ANLN could be restrained by elevating miR-30a-5p expression (Figures 5(d) and 5(e)). Altogether, miR-30a-5p could restrain cell processes of LUAD through mediating ANLN.

## 4. Discussion

It has been proven that miRNAs are involved in all stages of lung cancer, including initiation and progression [25]. Here is some compelling evidence. miR-593-5p restrains proliferation and migration of LUAD by targeting ICAM-1 [26]. circCRIM1 suppresses LUAD tumorigenesis through modulating miR-125b-5p/BTG2 axis [27]. miR-210 hastens tumorigenesis of LUAD cells through modulating lysyl oxidase like-protein 4 [28]. However, contribution of miRNA in the molecular mechanism of LUAD progression has not been fully clarified.

Here, we determined evidently d activated ANLN in LUAD tissues via bioinformatics analysis. Recently, many studies have documented that ANLN is crucial to the growth of cancer cells. For example, miR-497 suppresses cancer phenotypes of nasopharyngeal carcinoma through targeted regulation of ANLN and HSPA4L [23]. ANLN blocks cells in the G2/M phase in bladder urothelial carcinoma [29]. Especially, several studies focused on its effects on LUAD cell behaviors. For example, Xu and his colleagues demonstrated that enhancing the expression of ANLN in LUAD cells resulted in promoting cell migratory, invasive abilities as well as EMT progress [13]. For another study published in 2005, the molecular mechanisms of ANLN on promoting LUAD cell invasion and migration were described, in which ANLN-RHOA complex was elaborated [11]. Likewise, our data illustrated considerably stimulated ANLN in LUAD. Overexpressed ANLN hastened cell processes of LUAD. In conclusion, ANLN upregulation is a prerequisite for lung and bladder cancer progression.

RETRACTED

It has been reported on the relationship between ANLN and miRNA. For example, Wang et al. reported that ANLN-induced upregulation of EZH2 could promote the progression of pancreatic cancer [30]. Idichi et al. reported that the downregulation of ANLN by tumor suppressor miR-217 could inhibit the invasiveness of cancer cells in pancreatic ductal adenocarcinoma [24]. On this basis, this study revealed that miR-30a-5p may modulate ANLN in LUAD. Inactivated miR-30a-5p was discovered in different types of cancer including breast cancer [31], lung squamous cell carcinoma [32], oral carcinoma [33], and clear cell renal cell carcinoma [34] and could work as a cancer suppressor. The present investigation illustrated evidently restrained miR-30a-5p in LUAD and its targeting ANLN. qRT-PCR and WB illuminated that miR-30a-5p constrained ANLN in LUAD. At last, cell functional experiments indicated that upregulating miR-30a-5p could reverse the promoting effect of ANLN upregulation on cell progression in LUAD. Overall, these results identified that miR-30a-5p mediated ANLN to inhibit LUAD cell progression.

Despite all findings above, this investigation is still limited. The *in vivo* function of miR-30a-5p/ANLN in LUAD has not been further investigated due to a lack of time. Potential mechanisms still need to be researched, and more discussions can be performed to fully understand the miR-30a-5p/ANLN axis in LUAD.

All in all, miR-30a-5p restrained the development of LUAD through downregulating the expression of ANLN resulting in poor prognosis of LUAD patients, which revealed the potential role of the miR-30a-5p/ANLN axis in LUAD. These results can provide potential biomarkers for prognosis evaluation and treatment intervention of LUAD.

RETRACTED

## Figures and Tables

**Figure 1:** Activated ANLN in LUAD indicates poor prognosis. (a) Volcano plot of differential mRNAs in the TCGA-LUAD dataset (red: upregulated, green: downregulated). (b) Violin plot of expression of ANLN (blue: normal group, orange: tumor group). (c) Survival curves show the association between ANLN expression and prognosis (red: highly expressed group, blue: lowly expressed group). (d) Violin plot showed correlations between different clinicopathological features and ANLN expression. (e) and (f) ANLN mRNA and protein levels in A549, PC9, H1299, and H1975 cells were upregulated; ^∗^ represents *p* < 0.05, ^∗∗∗^represents *p* < 0.01, and ^∗∗∗∗^ represents *p* < 0.0001.

**Figure 2:** ANLN promotes the progression of LUAD. (a) The transfection efficiency of ANLN was relatively high in LUAD cell line A549. (b) The proliferative ability of A549 cells was significantly increased and decreased after overexpressing and silencing ANLN, respectively. (c) and (d) The invasive (100×) and migratory abilities (40×) of A549 cells were markedly increased and decreased after overexpressing and silencing ANLN, respectively; ^∗^ represents *p* < 0.05.

**Figure 3:** Low level of miR-30a-5p in LUAD. (a) Volcano plot of differential miRNAs (red: upregulated, green: downregulated). (b) Venn diagram of predicted miRNAs of ANLN and differential miRNAs. (c) Among 3 differential miRNAs, miR-30a-5p displayed the highest Pearson negative correlation with ANLN. (d) Boxplot of miR-30a-5p expression (green: normal, red: tumor). (e) qRT-PCR detection result; ^∗^ represents *p* < 0.05.

**Figure 4:** miR-30a-5p restrains ANLN in LUAD cells. (a) Predicted complementary binding sequences. (b) The luciferase activity of cells after transfection. (c) and (d) After transfection with miR-30a-5p mimic, mRNA and protein level of ANLN were significantly downregulated; ^∗^ represents *p* < 0.05.

**Figure 5:** Upregulating miR-30a-5p counteracts promoting effect of ANLN upregulation on biological behaviors of LUAD cells. (a) and (b) The mRNA and protein levels of ANLN in A549 cells in different transfection groups. (c) Upregulating miR-30a-5p counteracted promoting effect of overexpressed ANLN on cancer cell proliferation. (d) and (e) Upregulating miR-30a-5p counteracted promoting effect of overexpressed ANLN on the invasive (100×) and migratory abilities (40×) of A549 cells; ^∗^ represents *p* < 0.05.

**Table 1:** qRT-PCR primer sequences.

Gene	Primer sequences (5′→3′)
miR-30a-5p	F: TACGGATCCCCTTCATCTTACTTTTTTCCCCCAA
	R: ATCGCTAGCGAAACTAGAAGCTCGGTGATGAATA

U6	F: CTCGCTTCGGCAGCACA
	R: AACGCTTCACGAATTTGCGT

ANLN	F: CAAGATGTATCCAATGACT
	R: TGACTGAAGAATGAATGTT

*β*-Actin	F: CATGTACGTTGCTATCCAGGC
	R: CTCCTTAATGTCACGCACGAT

RETRACTED

## Data Availability

No data were used to support this study.

## References

[1] Hirsch F. R., Scagliotti G. V., Mulshine J. L. (2017). Lung cancer: current therapies and new targeted treatments. *Lancet*.

[2] Lavin Y., Kobayashi S., Leader A. (2017). Innate immune landscape in early lung adenocarcinoma by paired single-cell analyses. *Cell*.

[3] Siegel R. L., Miller K. D., Jemal A. (2018). Cancer statistics, 2018. *CA: a Cancer Journal for Clinicians*.

[4] Field C. M., Alberts B. M. (1995). Anillin, a contractile ring protein that cycles from the nucleus to the cell cortex. *The Journal of Cell Biology*.

[5] Oegema K., Savoian M. S., Mitchison T. J., Field C. M. (2000). Functional analysis of a human homologue of the drosophila actin binding protein anillin suggests a role in cytokinesis. *The Journal of Cell Biology*.

[6] Xia L., Su X., Shen J. (2018). <em>ANLN </em>functions as a key candidate gene in cervical cancer as determined by integrated bioinformatic analysis. *Cancer Management and Research*.

[7] Sadi A. M., Wang D. Y., Youngson B. J. (2011). Clinical relevance of DNA microarray analyses using archival formalin-fixed paraffin-embedded breast cancer specimens. *BMC Cancer*.

[8] Olakowski M., Tyszkiewicz T., Jarzab M. (2009). NBL1 and anillin (ANLN) genes over-expression in pancreatic carcinoma. *Folia Histochemica et Cytobiologica*.

[9] Tamura K., Furihata M., Tsunoda T. (2007). Molecular features of hormone-refractory prostate cancer cells by genome-wide gene expression profiles. *Cancer Research*.

[10] Weinberger P., Ponny S. R., Xu H. (2017). Cell cycle M-phase genes are highly upregulated in anaplastic thyroid carcinoma. *Thyroid*.

[11] Suzuki C., Daigo Y., Ishikawa N. (2005). ANLN plays a critical role in human lung carcinogenesis through the activation of RHOA and by involvement in the phosphoinositide 3-kinase/AKT pathway. *Cancer Research*.

[12] Long X., Zhou W., Wang Y., Liu S. (2018). Prognostic significance of ANLN in lung adenocarcinoma. *Oncology Letters*.

[13] Xu J., Zheng H., Yuan S. (2019). Overexpression of ANLN in lung adenocarcinoma is associated with metastasis. *Thoracic Cancer*.

[14] Li H. Y., Liang J. L., Kuo Y. L. (2017). miR-105/93-3p promotes chemoresistance and circulating miR-105/93-3p acts as a diagnostic biomarker for triple negative breast cancer. *Breast Cancer Research*.

[15] Yu Y., Yin W., Yu Z. H. (2019). miR-190 enhances endocrine therapy sensitivity by regulating SOX9 expression in breast cancer. *Journal of Experimental & Clinical Cancer Research*.

[16] Ibuki Y., Nishiyama Y., Tsutani Y. (2020). Circulating microRNA/isomiRs as novel biomarkers of esophageal squamous cell carcinoma. *PLoS One*.

RETRACTED

[17] Zhou L., Jia S., Ding G. (2019). Down-regulation of miR-30a-5p is associated with poor prognosis and promotes chemoresistance of gemcitabine in pancreatic ductal adenocarcinoma. *Journal of Cancer*.

[18] Wang Y., Chen L., Guo Y. L., Li G. H., Ying C. C. (2019). Effect of long-chain non-coding RNA-AC024560.2 on proliferation and invasion of prostate cancer cells by targeted regulation of miR-30a-5p. *Zhonghua Yi Xue Za Zhi*.

[19] Li J., Zhao L. M., Zhang C. (2020). The lncRNA FEZF1-AS1 promotes the progression of colorectal cancer through regulating OTX1 and targeting miR-30a-5p. *Oncology Research*.

[20] Song F., Xuan Z., Yang X., Ye X., Pan Z., Fang Q. (2020). Identification of key microRNAs and hub genes in non-small-cell lung cancer using integrative bioinformatics and functional analyses. *Journal of Cellular Biochemistry*.

[21] Kumarswamy R., Mudduluru G., Ceppi P. (2012). MicroRNA-30a inhibits epithelial-to-mesenchymal transition by targeting Snai1 and is downregulated in non-small cell lung cancer. *International Journal of Cancer*.

[22] Li X., Liu J., Liu M., Xia C., Zhao Q. (2020). The Lnc LINC00461/miR-30a-5p facilitates progression and malignancy in non-small cell lung cancer via regulating ZEB2. *Cell Cycle*.

[23] Wang S., Mo Y., Midorikawa K. (2015). The potent tumor suppressor miR-497 inhibits cancer phenotypes in nasopharyngeal carcinoma by targeting ANLN and HSPA4L. *Oncotarget*.

[24] Idichi T., Seki N., Kurahara H. (2017). Regulation of actin-binding protein ANLN by antitumormiR-217inhibits cancer cell aggressiveness in pancreatic ductal adenocarcinoma. *Oncotarget*.

[25] Inamura K., Ishikawa Y. (2016). MicroRNA in lung cancer: novel biomarkers and potential tools for treatment. *Journal of Clinical Medicine*.

[26] Zhang H. B., Shen B., Ma Z. C., Xu Y. Y., Lou Y. L., Chen M. (2020). MiR-593-5p inhibited proliferation and migration of lung adenocarcinoma by targeting ICAM-1. *European Review for Medical and Pharmacological Sciences*.

[27] Zhang S. J., Ma J., Wu J. C., Hao Z. Z., Zhang Y. A., Zhang Y. J. (2020). Circular RNA circCRIM1 suppresses lung adenocarcinoma cell migration, invasion, EMT, and glycolysis through regulating miR-125b-5p/BTG2 axis. *European Review for Medical and Pharmacological Sciences*.

[28] Xie S., Liu G., Huang J., Hu H. B., Jiang W. (2019). miR-210 promotes lung adenocarcinoma proliferation, migration, and invasion by targetinglysyl oxidase-like 4. *Journal of Cellular Physiology*.

[29] Zeng S., Yu X., Ma C. (2017). Transcriptome sequencing identifies ANLN as a promising prognostic biomarker in bladder urothelial carcinoma. *Scientific Reports*.

RETRACTED

[30] Wang A., Dai H., Gong Y. (2019). ANLN-induced EZH2 upregulation promotes pancreatic cancer progression by mediating miR-218-5p/LASP1 signaling axis. *Journal of Experimental & Clinical Cancer Research*.

[31] Li L., Kang L., Zhao W. (2017). miR-30a-5p suppresses breast tumor growth and metastasis through inhibition of LDHA-mediated Warburg effect. *Cancer Letters*.

[32] Chen C., Tang J., Xu S., Zhang W., Jiang H. (2020). miR-30a-5p inhibits proliferation and migration of lung squamous cell carcinoma cells by targeting FOXD1. *BioMed Research International*.

[33] Ruan P., Tao Z., Tan A. (2018). Low expression of miR-30a-5p induced the proliferation and invasion of oral cancer via promoting the expression of FAP. *Bioscience Reports*.

[34] Chen Z., Zhang J., Zhang Z. (2017). The putative tumor suppressor microRNA-30a-5p modulates clear cell renal cell carcinoma aggressiveness through repression of ZEB2. *Cell Death & Disease*.

